# HIV-1 associated dementia: symptoms and causes

**DOI:** 10.1186/1742-4690-3-28

**Published:** 2006-05-19

**Authors:** Mohammad Ghafouri, Shohreh Amini, Kamel Khalili, Bassel E Sawaya

**Affiliations:** 1 Department of Neuroscience, Center for Neurovirology, Temple University School of Medicine, Pennsylvania 19122, USA; 2 Department of Biology, College of Science and Technology, Temple University, Philadelphia, Pennsylvania 19122, USA

## Abstract

Despite the use of highly active antiretroviral therapy (HAART), neuronal cell death remains a problem that is frequently found in the brains of HIV-1-infected patients. HAART has successfully prevented many of the former end-stage complications of AIDS, however, with increased survival times, the prevalence of minor HIV-1 associated cognitive impairment appears to be rising among AIDS patients. Further, HIV-1 associated dementia (HAD) is still prevalent in treated patients as well as attenuated forms of HAD and CNS opportunistic disorders. HIV-associated cognitive impairment correlates with the increased presence in the CNS of activated, though not necessarily HIV-1-infected, microglia and CNS macrophages. This suggests that indirect mechanisms of neuronal injury and loss/death occur in HIV/AIDS as a basis for dementia since neurons are not themselves productively infected by HIV-1. In this review, we discussed the symptoms and causes leading to HAD. Outcome from this review will provide new information regarding mechanisms of neuronal loss in AIDS patients.

## Definition and causes

Dementia cannot be considered as a disease by itself but it is the term used to describe a set of symptoms resulting from damages and disorders affecting the brain. These symptoms can be caused by a multitude of diseases and depend upon the specific brain regions affected. These symptoms appear as a variety of cognitive, behavioral, affective, motor, and psychiatric disorders. Dementia can be caused by a variety of diseases, known as neurodegenerative diseases resulting from protein aggregation in the brain [1]. These diseases include Alzheimer's, Lewy bodies, Huntington and Parkinson [1]. Infectious diseases affecting the central nervous system (CNS) may lead to dementia. These infections can be caused by different agents such as: abnormal protein in prion diseases (Creutzfeldt-Jakob disease), bacteria in syphilis and borrelia, parasites in toxoplasmosis, cryptococcosis and neurocysticercosis [2], however viral agents are the leading cause of infection related dementia. Among the viruses infecting the brain, human immunodeficiency virus type 1 (HIV-1) is the most common cause of dementia, other CNS viral infection implying herpes simplex virus type I, Varicella zoster virus, cytomegalovirus, Epstein-Barr virus cause encephalitis and severe brain dysfunction. The collection of viral agent infecting the CNS and producing viral encephalitis includes also arboviruses, rabies viruses, polyomaviruses and enteroviruses [3]. Finally, dementia could also be caused by vascular disorders (e.g. multiple-infarct dementia), drug addiction, hydrocephalus, and injury or brain tumors [4,5]. Despite the variability of symptoms with the disease causing dementia there is overlap, potentially because of the involvement of common neural pathways and the nature of the damage. However, the time of appearance, the severity, and type of symptoms allow, in most cases, to help making the distinction between diseases. There are however cases of coexistence of clinical and/or pathological features where more than one disease is manifested in one individual, and which might be due to co-occurrence of common diseases within the individual [6]. In elderly populations, Alzheimer's disease is the most frequent cause of dementia, while neuroAIDS is the major cause of dementia in younger population (less than 60 years old). In the United States, HIV-1 infection is the most common cause of dementia in young adults [7,8]. Since many diseases and viral infection lead to dementia, we focused our review on HIV-1 associated dementia, its symptoms and causes.

## Neuropathology of AIDS

HIV-1 is the causative agent of acquired immunodeficiency syndrome (AIDS), which is a multi-system disorder including the CNS. Neurological impairment affects approximately 60% of HIV-infected patients [9]. HIV-1 enters the CNS at the early phase of infection [10], persists in that system for decades and induces multiple symptoms of motor, cognitive dysfunction and behavioral changes. Many factors can contribute to the neuropathology of AIDS, particularly opportunistic brain infections such as cryptococcus, Toxoplasma gondii, JC virus, cytomegalovirus, Epstein-Barr virus, Varicella zoster virus, and human herpes virus type 6 [2]. In the absence of opportunistic infections, major clinical symptoms include impaired short term-memory coupled with reduced ability of mental concentration, leg weakness, slowness of hand movement and gait as well as depression [11,12]. These symptoms are often accompanied by behavioral symptoms such as personality changes, apathy and social withdrawal. The terms AIDS dementia complex (ADC), and HIV-1 associated dementia (HAD), are used to describe these neurological and psychiatric symptoms caused by HIV-1 infection [11,12]. An effective therapy for HIV/AIDS became available in 1995, generally known as highly active antiretroviral therapy (HAART). This therapy consists of a combination of at least three drugs blocking different aspect of viral replication, markedly reverse transcriptase inhibitors and protease inhibitors. HAART has the capability of restoring immune function; suppressing viral replication to nearly undetectable level, consequently ameliorating HIV related symptoms in the CNS and preventing opportunistic conditions. Before the introduction of HAART, nearly 30% of the infected population developed HAD at the late stage of HIV/AIDS. With the use of HAART this rate is reduced to 10% [13]. However, a more subtle form of CNS dysfunction, known as minor cognitive motor disorder (MCMD), has become more common in HIV patients [14]. In this condition, memory loss and the reduction of cognitive and computational functions are much less pronounced. Recently it has been estimated that nearly 30% of adults infected with HIV are affected by MCMD. However, HAD is far from being controlled by HAART; in the setting of HAART the HIV-1 infection become chronic and recent studies show a rise in the incidence of the HAD [3], it is noteworthy that HAART is not designed to target the inflammatory cascade underlying the HAD. In addition some of the HIV-1 infected population develop resistance against HAART and an important fraction of AIDS patients, especially in developing countries, have not access to HAART. In the United States, HIV-1 infection is the most common cause of dementia in young adults [7,8].

The HIV-1 associated neuropathology is characterized by the infiltration of macrophages into the CNS; the formation of microglial nodules; and multinucleated giant cells which result possibly from virus-induced fusion of microglia and/or macrophages in central white and deep gray matter; astrocyte activation and damage; neuronal loss particularly in hippocampus, basal ganglia and caudate nucleus. In addition, a variable degree of white matter pathology with evidence of broad range of myelin damage ranging from pallor to widespread breakdown and loss leading to accumulation of lipid macrophages in extreme cases, with axonal damage in the latter cases, and the presence of HIV-1 in the cerebral spinal fluid (CSF) has been reported [13,15]. These neuropathological consequences of infection are collectively termed HIV-1 associated encephalitis (HIVE).

Clinical observations, using MRI, confirm that HIV infection is associated with progressive cortical atrophy within the gray and white matter in the brain, particularly in the later stage of the disease [16-19]. These studies report a correlation between the deterioration of cognitive function and the reduction in volume of certain brain structures including the basal ganglia and caudate nucleus. Volumetric MRI analysis has shown that cortical atrophy associated with HIV infection might be caused by neuronal loss and demyelination. The degree of atrophy is correlated to the degree of cognitive motor dysfunction in both cross-sectional and longitudinal cohorts [16,19,20]. Quantitative MRI shows a correlation between cerebral atrophy and neuropsychological performance. Over time, the correlation persists between an increase in atrophy and worsening in certain cognitive functions [16].

## Viral entry and replication

HIV-1 targets the lymphoid and nervous systems by infecting cells containing major HIV-1 receptors, CD4 and CD8, and various chemokine receptors considered as HIV-1 co-receptors. These receptors help the attachment of the virus to the cell and the fusion of their membrane resulting in the entry of the virus into the cell [21]. HIV-1-specific CD4^+ ^helper T lymphocytes and CD8^+ ^cytotoxic T lymphocytes have been detected within 4-6 weeks after HIV-1 inoculation [22]. Infected CD4^+ ^T cells and monocytes, which circulate in the blood, are the potential source of CNS infection [14]. The mechanisms of entry of these cells into the CNS are discussed in the next section. Among the chemokine receptors expressed on human cells, CXCR4 appears to be the most important for HIV-1 entry into lymphocytes and CCR5 for monocytes, macrophages and microglia [23]. Because of the variability of HIV-1 phenotypes, these strains of virus are defined by their usage of the CCR5 or CXCR4 co-receptors, and designated as R5- and X4- viruses respectively [23]. Following entry into the cell, the virus undergoes reverse transcription of its RNA genome to form a double-stranded DNA, a pre-integration complex of viral DNA with integrase and other viral protein including Vpr and matrix protein is transported to the nucleus. The pre-integration complex facilitates the integration of the HIV-1 DNA genome into host chromatin. The integration of viral DNA into the host cell genome generates the provirus that allows the production of HIV-1. In addition, high levels of viral DNA remain non-integrated in the nucleus and are capable of directing expression of viral transcript [24-26]. The generation of infectious virus particles involves the production of viral transcripts and proteins and viral assembly, release and maturation. During the production phase, first the vial regulatory factors Nef, Tat and Rev are generated, and viral structural proteins and the RNA genome are produced in a later phase. In the assembly phase, Gag and Gag-Pol Polyproteins, envelope proteins and viral RNA genomes are assembled into immature virus particles at the cell membrane and released from the host cell. The cleavage of Gag and Gag-Pol Polyproteins by the HIV-1 protease results in the production of mature virus [27-29].

The intracellular environment plays a major role in HIV-1 virus replication [30]. HIV-1 infected cells are classified as highly active producers and low or non-producers of viruses, known as "productive" and "restricted" infection, respectively. Both types of infections occur in the CNS. Productively infected cells support productive viral replication and participate in the transmission of the infection and the rapid evolution of viral genome in the human host and die ultimately. Restricted infection is only detectable by highly sensitive methods showing the presence of HIV-1 DNA or RNA. However, in the absence of structural viral protein expression, it has been reported that accessory/regulatory protein such as Rev and Nef have been expressed [31,32]. Restrictedly infected cells are permissive to infection by HIV-1 strains but are refractory to efficient virus expression, they restrict the HIV-1 replication and survive as virus reservoir in which replication-competent viral genome persists. The restricted infection implies that efficient HIV-1 replication might be blocked at different stage of virus life cycle, including virus entry, reverse transcription, nucleo-cytoplasmic HIV-1 RNA transport, translation of viral DNA, and maturation of progeny virion. Studies of different astrocytes cell lines, which are known to be non-productively infected, demonstrated a cytoplasmic presence of Rev up to seven time more elevated than in productively infected cells [33,34]. These observations lead to the hypothesis that restricted HIV-1 production in astrocyte may be partly due to a cell determined block in nucleo-cytoplasmic Rev shuttling causing the nuclear retention of Rev-dependent HIV-1 mRNA classes where they are degraded [35,32]. Changes in cell environment, like the elevation in the level of cytokines such as TNF-α and IL-1β, might reactivate virus production [10,36].

## Neuroinvasion of HIV-1

The role of blood-brain barrier (BBB), which is a continuous cellular layer of tightly linked brain microvascular endothelial cells, is to separate the CNS from the periphery (Figure 1). The BBB is selectively permeable and regulates the trafficking of cells and substances between the brain parenchyma and the bloodstream [14,15]. The CSF is also separated from the periphery by the blood-CSF barrier of the choroids-plexus epithelium. In order to enter the brain, HIV-1 must cross the BBB using mechanisms that remain unclear. Numerous studies have used animal models and *in vitro *experimentation to understand the mechanisms of HIV-1 introduction into the CNS through BBB [14]. The generally accepted model, with most compelling evidence, is the "Trojan Horse hypothesis" [37,38]. According to this model, HIV-1 and other lentiviruses enter the CNS as a passenger in cells trafficking to the brain (Figure 1). Many CD4+ cells, such as T cells and monocytes are infected by HIV-1, these cells circulate in the blood and can cross the BBB and propagate the infection within the CNS [37]. This model was confirmed by *in situ *hybridization and immunohistochemical analysis that brought evidence of virus accumulation in perivascular regions [39-41]. Though BBB abnormalities due to HIV-1 infection have been observed, however, the mechanisms of endothelial cells infection and the expression of conventional HIV receptors in these cells remain a controversial issue. Although some studies suggest that human brain microvascular endothelial cells lack CD4 receptors [42], other studies have found that CD4 was expressed in isolated endothelial cells and microvessels of HIV-1 infected children's brains [43,44], moreover the expression of HIV-1 co-receptors such as CCR5 and CXCR4 have also being reported on isolated primary human brain's microvascular endothelial cells [45]. An alternative hypothesis of HIV-1 neuro-invasion proposes the entry of free HIV-1 by migration between or, transcytosis of endothelial cells [10,14,46,47]. Theoretically all the main cell types of the CNS, astrocytes, oligodendrocytes, neurons, perivascular macrophage and microglia, can be infected by HIV-1 since they possess the receptors and/or co-receptors for HIV-1 entry, but only the latter two are the most commonly infected cells by HIV-1 [14].

**Figure 1:** HIV-1 neuroinvasion. 1) According to the "Trojan Horse hypothesis" entry of HIV-1 into the brain takes place by the migration of infected monocytes which differentiate into perivascular macrophage. 2) The passage of infected CD4^+ ^T cells can be another source of infection in the brain. Other probable causes of CNS infection might be: 3) the direct entrance of the virus or 4) entrance of HIV-1 by transcytosis of brain microvascular endothelial cells. Once the virus is in the brain it infects productively macrophages and microglia. Astrocyte infection is known to be restricted. The infection of oligodendrocytes and specially neurons is questionable.

### Macrophage and microglia

Perivascular macrophage, microglia, and astrocytes are the cells coming into direct contact with infected cells in perivascular region. The two first types of cells are the resident immunocompetent cells of the brain and their major role is to respond to all types of insults. Peripheral macrophage population is replenished through the lifespan with a relatively fast turnover, probably because of its proximity to the interface with the periphery. This replenishment that takes place by the migration of monocytes into the CNS has the side effect of opening the door to the intracellular pathogen. As the monocytes take residency in the CNS they differentiate into macrophages. Microglia and monocyte-derived macrophage are considered to be the main sources of productive HIV-1 infection in the brain [48,49]. One of the characteristics of HIVE is the presence of multinucleated giant cells expressing CD4. These cells are assumed to be infected monocytes differentiated into macrophage after entering the brain or arising from the fusion of infected microglia [50]. It has been shown that in the primate Simian Immunodeficiency Virus (SIV) model the spread of the virus from perivascular cells to the parenchymal microglia does not occur [51], however this issue remains controversial and has not been confirmed for SIV and HIV-1. In contrast, many studies suggest the opposite for HIV-1. Immunostaining has revealed HIV-1 infection of parenchymal microglia, in some cases the infection is widespread, but in other cases it is restricted to the perivascular compartment [52]. It is not clear whether the HIV-1 immunopositive microglia consists of an influx of infected cells from the blood or results from long-term infection in the CNS. In-vitro studies have demonstrated that HIV-1 replication takes place in primary microglia isolated from adults [53,54], infants [55], and fetal brain [56,57]. HIV-1 infection in Microglia can be associated with cytopathology, including the formation of syncytia [54]. The study of the course of HIV-1 infection in purified primary cultures of human microglia shows that productive infection was more readily established by R5-tropic strains of HIV-1 than by an X4-tropic strain [55]. Microglial cells similar to macrophage express, CD4/CCR5, major receptors/co-receptors used by HIV-1 [58-60]. Other chemokine receptors, e.g. CCR3, CCR2b, CCR8, CXCR6, and CX3CR1, are also expressed by these cells but less efficiently used by HIV-1 [60,61]. I*n vitro *studies have shown that long-lived mixed microglial cultures isolated from human brain, when infected with R5 HIV-1, retain replication competent viruses for up to 2.5 months with low level virus replication, providing an activating condition can result in productive virus replication [62].

### Astrocytes

Astrocytes do not have the CD4 receptor, which plays an important role in the infection of immune system cells, but they express CXCR4 and possibly other HIV-1 co-receptors including CCR5 [32]. However, several studies have reported the infection of astrocytes by HIV-1 although the mechanisms of viral attachment to astrocytes remain unclear. Immunopositivity of astrocytes for HIV-1 structural proteins has occasionally been reported [35]. However, *in situ *hybridization, or *in situ *PCR have revealed the presence of HIV-1-specific nucleic acids in astrocytes [40,63,64]. Other studies reported the presence of the viral DNA and HIV-1 Nef protein in astrocytes [65].

HIV-1 infection was studied using primary human fetal astrocytes and tumor derived cell lines, several HIV-1 isolates, namely X4-using T-cell line adapted (NL4-3, 1 MB, SF2), R5-using, macrophage tropic (JR-FL, SF162) strains and primary isolates from blood [32,66,67]. The participation of astrocytes in productive infection has not been reported, though virus production in persistently infected cells can be transiently activated by the treatment with inflammatory cytokines [32,66,67].

### Oligodendrocytes

I*n vivo*, Oligodendrocytes infection by HIV-1 remains controversial. While some studies have detected viral nucleic acids by in situ PCR [63,64], other studies have reported the absence of HIV-1 markers in oligodendrocytes [33]. I*n vitro *studies, using human oligodendrocytes indicates restricted infection by R5 and X4 strains of the virus [68]. Some studies have reported a reduced expression of specific oligodendrocyte markers, such as MBP and CNPase, in mice expressing HIV-1 Nef [69]. Oligodendrocytes do not possess CD4 receptors and the mechanisms of their potential infection remain unclear.

### Neurons

Most studies have indicated an absence of *in vivo *infection in neurons, however a few studies have reported the presence of HIV-1 DNA and proteins in neurons [63,64]. It has been suggested that the detection of infected neurons in the brain might be complicated by the loss of the infected neuronal populations [14]. I*n vitro *studies have reported restricted infection of primary neurons [70], and neuronal cell lines by X5 and R4 viruses [71,72].

## Mechanisms of neurodegeneration in HIV-associated dementia

The absence of significant neuronal infection by HIV-1 contrasts with the extensive neuropathological damage observed in HAD, therefore different mechanisms involving the HIV-1 infection of perivascular macrophages, microglia, and possibly astrocytes might play the principal role in neuronal injury and the disruption of normal neurological function. The neuronal injury can result from a direct mechanism by interaction with viral proteins, such as gp120, Tat (Transcriptional transactivator) and Vpr (viral protein R) produced by infected cells, or by an indirect effect resulting from the inflammatory process involving activated monocytes, macrophages and astrocytes (Figure 2).

**Figure 2:** Mechanism of neuropathogenesis. Two components of this mechanism are: A) the direct effect of the HIV-1 infection, including HIV-1 proteins and B) the indirect consequence of infection comprising the secretion of cytokines and neurotoxins. The infected macrophages and microglia participate actively in the neurodegeneration by: 1) shedding viral proteins and 2) releasing significant amount of cytokines and neurotoxins into the CNS. 3) Tat and TNF-α contribute to the disruption of the blood brain barrier, which in turn become more permeable to infected monocytes and cytokines present in the periphery. The secreted pro-inflammatory cytokines activates 4) microglia and 5) astrocytes which in turn secrete neurotoxins, moreover the alteration of astrocytes function results in an increase in the level of neurotoxicity in the brain. 6) Multifactorial neuronal injury: neurotoxins released from several sources, as the direct and indirect consequences of HIV-1 infection, lead to neuronal injury.

### HIV-1 Tat

The viral protein Tat, which is mainly active in the nucleus, was shown to be secreted at high-level *in vitro*. Secreted Tat can cause direct or indirect injury to neurons, therefore it has been suggested that Tat contributes to HAD neuropathogenesis [73]. The neurotoxicity of Tat involves prolonged increase in intracellular calcium followed by an increase of reactive oxygen species and caspase activation of apoptotic pathway [73,74], in addition it has been shown that the up-regulation of caspase-8 by HIV-1 Tat expression in CD4 T cell lines may contribute to the increased apoptosis and sensitivity to apoptotic signals [75]. Tat is shown to alter the expression distribution of tight junction proteins, claudin-1 and claudin-5 in cerebral microvascular endothelial cells [76]. By affecting endothelial permeability, Tat contributes to the disruption of the BBB that leads to infiltration of inflammatory cells into the CNS [76,77]. Further, Tat participates in the HAD associated inflammatory cascade by promoting TNF-α and interleukin IL-1 production by monocytes and macrophages, and stimulates the production of several cytokines and chemokines, including IL-8, RANTES, MCP-1 and TNF-α in astrocytes, which leads to neurotoxicity [73].

### HIV-1 Vpr

The regulatory protein Vpr might also be a player in the direct mechanism of neuronal damage (reviewed in [78]). Vpr has been found in the CSF of HAD patients [79]. Vpr induces cell cycle arrest at G2/M phase, which leads to cell death [80], a recent model of Vpr mediated induction of apoptosis, in CD4+ cells, proposes that Vpr expression activates cancer-associated protein BRCA1 and up-regulates the expression of DNA damage-45 protein α (GADD45α) [81]. It has been reported that Vpr also alters mitochondrial permeability, which can cause cytochrome *c *release and eventually lead to apoptosis [82], however this issue needs to be confirmed. Furthermore, another study of Vpr-mitochondria interaction has shown that Vpr targets HAX-1, an antiapoptotic mitochondrial protein, Vpr associates physically to that protein and Vpr over-expression leads to dislocation of HAX-1 from its normal mitochondrial residence and causes mitochondrial instability and apoptosis [83]. Recent studies have demonstrated that both intracellular and extra cellular Vpr can induce apoptosis of human neuronal-precursor cells and mature, differentiated neurons by increasing the activation of caspase-8 [84]. Finally, Tat and Vpr mediated-apoptosis could increase significantly by co-exposure of cells to ethanol [84,85].

### HIV-1 gp120

HIV-1 envelope glycoprotein gp160 is shown to have neurotoxic effect. This protein can be cleaved into two products that remain non-covalently associated: gp120 and gp41. The soluble viral envelope protein gp120, which is released in large quantities by HIV infected cells, might be involved in neuronal injury. The toxic effect of gp120 on neuronal population was demonstrated by many studies [86,87], dopaminergic neurons might be more susceptible to gp120 neurotoxicity [88]. It has been shown that transgenic mice overexpressing gp120 had neuropathological features similar to abnormalities in brains of HAD patients [89]. Neurodegeneration induced by gp120 can be direct through interaction with NMDA (N-Methyl-D-Aspartate) receptor or indirect by interaction with chemokine receptors [90,91]. Further, it has been shown that the presence of p53 is essential for gp120-induced neuronal apoptosis [92]. Furthermore, both gp120 and Tat have been shown to disrupt neuronal calcium homeostasis by perturbing calcium-regulating systems in the plasma membrane and endoplasmic reticulum, which leads to neuronal death [93]. Recently, it has been described that SDF-1α and gp120 induced a similar level of neuronal apoptosis, but by activating different intracellular pathways. SDF-1α enhanced NMDA activity indirectly *via Src *phosphorylation, whereas gp120 probably activated the NMDA receptor directly and phosphorylated JNK [94]. These results are in accord with other studies, where gp120 was shown to induce neuronal dysfunction and death through actions at p38 mitogen-activated protein kinase, while Tat kills neurons through actions that are independent of p38 or c-jun-N-terminal kinase mitogen-activated protein kinase, or through the concurrent activation of multiple pro-apoptotic pathways [95].

Some chemokine receptors are considered to act as a direct conduit for gp120 neurotoxicity, whereas others can have neuro-protective effects [49,87]. The role of CXCR4 in the gp120 mediated neurotoxicity can be direct, through the activation of neuronal receptors by gp120, or indirect through the stimulation of glial cells leading to release of neurotoxic factors. Several studies have shown that T tropic (X4) and dual tropic (X4/R5) gp120 induce apoptosis in primary neurons and in neuronal cell lines [96,97]. In contrast to the neuroprotective role of RANTES/CCL5 and MIP-1β against gp120, in mixed neurons/glial cultures, it has been shown that SDF-1α/CXCL2 not only failed to provide neuro-protection from gp120, but induced apoptosis in its absence [49]. Beside its direct neurotoxic effect, the viral protein gp120 has a significant role in the indirect mechanisms of neurodegenertion by acting on macrophages, microglia or astrocytes [87,96]. Gp120 interaction with astrocytes stimulates the inducible form of nitric oxide synthase and increases the release of arachidonic acid from astrocytes, which leads to the inhibition of glutamate uptake by astrocytes and neurons [98]. As a result the extracellular concentration of glutamate increases and could lead to neurotoxicity via activation of excitatory amino acid receptors on neurons [73]. By acting on monocytes and macrophages gp120 induces the production of TNF-α, IL-1 and arachidonic acid metabolites which are implicated in HIV-1 neuropathogenesis.

### HIV-1 associated chemokines

The chemokines and their receptors are considered to be involved in the pathogenesis of a number of neurological diseases including HAD, multiple sclerosis, Alzheimer's disease, and prion infection. The over-expression of some chemokines in specific brain areas might contribute to the pathological condition. The chemokines and their receptors are the gate of entrance of HIV into the CNS [99]. Because of the alterations and abnormalities in the expression of chemokines and their receptors in the HIV infected CNS cells, and the role of chemokines in several neurodegenerative diseases, they have been the focus of attention in studies of HAD pathogenesis [100]. All members of the CXCR family are expressed, mainly by neurons, in the brains of individuals affected by HAD [101]. Semiquantitative immunohistochemical analysis of the brain of HIV-1 infected individual, investigating the expression of four HIV-1 co-receptors CCR2, CCR3, CCR5 and CXCR4 has shown that the hippocampal neurons were positive for CCR2, CCR3, and CXCR4 [102]. In other regions of the brain, neurons, as well as glial cells were positive for CCR2, CCR3, and CXCR4, whereas only primary microglial cells were positive for CCR5. The areas of highest expression seem to be subcortical regions and the limbic system. The role of limbic system in memory and other cognitive functions, and the presence of CXCR4 on a subpopulation of neuron from this system might explain cognitive and memory dysfunction in HAD. The presence of chemokines and chemokine receptors increases in the brain tissues of HIVE patients, particularly in areas of neuroglial reaction, where they might be involved in the recruitment of inflammatory infiltrates and formation of microglial nodules. The levels of expression of CCR1, CCR3, CCR5 and CXCR4 are especially elevated in the microglial nodules [59,103]. Moreover, CCR3 and CXCR4 are highly expressed in the pyramidal neurons of hippocampus, and in the enthorinal cortex for CCR3. Compared to AIDS patients without HAD, the brain tissue of patients with HAD shows an over-expression of CX_3_C chemokine, fractalkine/CX3CL1 [104,105]. The upregulation of fractalkine/CX3CL1 was found in neurons in brains of pediatric patients [104]. In contrast, fractalkine/CX3CL1 was found to be over-expressed in astrocytes in adult patients [105]. The level of chemokines in the CSF of HIV-infected patients with and without HAD has been determined in several studies. The results show that CSF chemokine concentration of MCP-1/CCL2, MIP-1α/CCL3, MIP-1β/CCL4, RANTES/CCL5, IL-8/CXCL8 and fractalkine/CX3CL1 is positively correlated with the severity of dementia and the viral load, indicating HIV induced brain damage. The role of CCR5, which is expressed by neurons, microglia and astrocytes in the brain, seems more controversial in the pathogenesis of HAD. The activation of CCR5 by RANTES or MIP-1α/β, in in-vitro studies, is shown to offer neuro-protection against gp120 induced apoptosis [87,106]. However, *in vitro *observations indicate that neuro-virulent strains of HIV are essentially M-tropic with increased affinity for CCR5 [107]. It has also been shown that CCR5 activation via its specific ligand induced apoptosis in neuroblastoma but not in fibroblast cell lines [108]. Therefore, it can be assumed that CCR5 might act as a death receptor in neurons and participate in HIV-1 induced neuropathology.

In brief, cognitive, motor decline and behavioral disorders in HAD can be explained by significant neuronal cell death that has been reported as a consequence of HIV-1 infection in the brain [109,110]. However, very few trace of infection has been found in neurons of HAD patients' brains. Therefore the neuronal loss might be caused by the release of neurotoxic factors by HIV infected microglia and astrocytes and/or by neurotoxic HIV-1 proteins.

### The inflammatory cascade

The indirect mechanisms of AIDS neuropathogenesis also include the effect of the inflammation resulting from the modification of extracellular secretory functions of microglia and brain macrophages and inflammatory cytokine production in the CNS (Figure 2). Following entry to the brain, monocytes, lymphocytes, activated macrophage, microglia and astrocytes release cytokines, reactive oxygen species, and other neurotoxins that disrupt normal cellular functioning, modify neurotransmitter action, and may lead to leukoencephalopathy and ultimately neuronal apoptosis [111,112]. Some of these neurotoxins include TNF-α, arachidonic acid, platelet activating factors (PAF), nitric oxide (NO), and quinolinic acid (QUIN). NO is synthesized by endothelial cells, macrophages and neurons and might be associated with the NMDA type glutamate associated neurotoxicity. A high level of inducible NO synthase has been found in the brain of HAD patients [113]. In HIV-1 patients who also are/were drug addicted (e.g. cocaine, heroine), a 40-fold increase in expression of NO synthase in neurons of temporal lobes was reported [114]. TNF-α is released by HIV-1 infected macrophage microglia and particularly affects oligodendrocytes [115]. It has been shown that TNF-α mRNA level in the subcortical regions of HAD patients' CNS are higher than in AIDS patients without neurological symptoms [116]. In addition, TNF-α can damage the BBB, as shown in an in-vivo model, which could facilitate entry into the brain of HIV-1 protein(s) and cytokines secreted in the periphery [117]. Not only the level of pro-inflammatory cytokines, such as TNF-α, IL-1 and IFN-γ, anti-inflammatory cytokines including TGF-β and IL-6, and soluble cytokine receptors is elevated in AIDS patients, but the cytokine production is correlated with the gravity of the neuropathology [118,119].

This review is a summary of some of the current data supporting both the direct and indirect mechanisms by which neuronal death may occur during infection with HIV-1. HAD is a complex phenomenon, which could be the result of several mechanisms caused by players using different pathways. Some of these players, mechanisms, and pathways were mentioned in this review and some of them are either un-identified or left out e.g. MCP-1, cellular proteins involved in the regulation of HIV-1 gene expression, Ca^++ ^induction, HIV-1 activated apoptotic programs (reviewed in [120]). Finally, more strategies are needed for treating or preventing HAD by targeting specific neurotoxic mechanisms used by the above-mentioned viral proteins.

## Competing interests

The author(s) declare that they have no competing interests.

## Authors' contributions

MG wrote the manuscript, SA and KK shared ideas and discussion, BES conceived of the plan for the manuscript and coordinated its preparation. All authors read and approved the final manuscript.
